# Single-Segment Lumbar Intervertebral Disc Nucleus Excision on the Stability of Lumbar Segmental Sagittal Plane

**DOI:** 10.1155/2022/5858257

**Published:** 2022-03-15

**Authors:** Xiaobiao Du, Weifeng Zhang, Guoshun Huang, Feng Han, Xia Li, Jingguo Li

**Affiliations:** ^1^Department of Orthopaedics, General Hospital of Tisco, Sixth Hospital of Shanxi Medical University, Taiyuan City 030003, China; ^2^Department of Orthopaedics, The Second Affiliated Hospital of Henan University of Science and Technology, Luoyang City 471000, China; ^3^Shanxi Cardiovascular Hospital, Taiyuan City 030002, China

## Abstract

At present, lumbar disc herniation has become a problem that plagues people's health, life safety, and social and economic development. Among them, the research of lumbar disc nucleus pulposus tissue is the focus of the treatment of lumbar disc diseases. At present, the treatment methods of lumbar disc herniation are divided into conservative treatment and surgical treatment, among which surgical treatment can be divided into open surgery and minimally invasive surgery. Surgical treatment to remove the nucleus pulposus from the disc by fenestration includes conventional ablation of the nucleus pulposus and microscopic lumbar discs. This treatment is effective, but it has a great impact on the stabilization mechanism of the spine, with large soft tissue damage and large blood loss, which can easily cause nerve damage and postdural adhesions. At the same time, single-segment lumbar discectomy has also been gradually applied to the treatment of this disease. Under this, this paper studies single-segment lumbar disc nucleus pulposus resection. The lumbar nucleus resection is performed in a single segment in the physiological load area, which can greatly ensure the stability of the sagittal plane of the lumbar spine. In order to better understand the postoperative rehabilitation and clinical effects of single-segment lumbar discectomy, as well as the changes in the sagittal plane of the lumbar vertebrae before and after the operation, so as to provide a reference for further improving the quality of life of patients, this paper uses questionnaire survey and data analysis methods. According to the results of the questionnaire survey, compared with other operations, single-segment lumbar discectomy is more stable in the sagittal plane of the lumbar spine within the physiological load range, and there is less displacement. The displacement may be caused or influenced by different kinds of factors such as heavy loads or manual labor. In addition, most patients have less abnormal pain after surgery, indicating that the surgery has a certain effect on the treatment of the disease, and there are fewer abnormalities after surgery.

## 1. Introduction

From the current point of view, due to various congenital or acquired factors, patients with lumbar disc herniation tend to be younger and younger. This disease is the most common clinical orthopedic disease, and it is affected by a variety of pathogenic factors, such as pain, swelling, and joint capsule stenosis. Patients with lumbar disc herniation are prone to systemic inflammation when the spine is injured. Studies have shown that the success rate of early results of lumbar discectomy is as high as 90%. However, as the postoperative follow-up time is prolonged, it may leave sequelae to the patient and affect certain parts of the body. Therefore, this article carried out a basic study on the effect of single-segment lumbar disc nucleus extraction on the stability of the lumbar segmental sagittal plane.

At present, many experts and scholars in the medical field have conducted related research on lumbar disc nucleus extraction. For example, Minli et al. analyzed the diagnostic value of magnetic resonance imaging in the diagnosis of intervertebral space infection after lumbar disc herniation and nucleus pulposus excision and found that the sensitivity of enhanced MRI in diagnosing intervertebral space infection was significantly higher than that of plain MRI. There is greater value in the analysis [1]. Long et al. believes that the application of three-dimensional reconstruction technology to lumbar intervertebral disc nucleus extraction can help the successful completion of the operation, help patients relieve the pain caused by the operation, and improve the symptoms of the disease [2]. Jiamei and Xiaojing proposed that timely rehabilitation care for patients with lumbar disc herniation who are undergoing nucleus pulposus treatment can reduce their pain and reduce lumbar spine function problems [3].

This article mainly discusses these aspects. First, the basic concepts and treatment methods of lumbar disc herniation are introduced in detail. Then, the nucleus pulposus of the lumbar intervertebral disc and its related research were discussed in detail. In addition, the study on the stability of lumbar spine segments is also described. Finally, in order to better understand the therapeutic effect of single-segment lumbar discectomy and its influence on the stability of the lumbar segmental sagittal plane, a questionnaire survey was launched, and the corresponding investigation results and analysis conclusions were drawn.

Although many experts and scholars in the medical field have conducted relevant research on the treatment of lumbar disc herniation, further research is needed on the stabilization mechanism of the postoperative spine. Therefore, this article conducts basic research on the stability of lumbar segmental sagittal plane by single-segment lumbar discectomy, which provides an important reference value for exploring the postoperative rehabilitation and clinical effects of patients and further improving the quality of life of patients.

## 2. Related Theoretical Overview and Research

### 2.1. Lumbar Disc Herniation and Treatments

From the current point of view, lumbar disc herniation is one of the most common diseases in the spine. With the development of society, the pressure on people's work and life is increasing, the population is aging, and the incidence of lumbar disc herniation is also increasing. It has become one of the main diseases that threaten human health and reduce the quality of life and has become one of the key diseases in clinical research of spinal surgery.

The epidemiological characteristics of the disease are as follows: the incidence of lumbar disc herniation is highest in the 4th and 5th lumbar vertebrae, the 5th lumbar vertebrae, and the sacral space. Young people are more likely to get this disease, while older people generally suffer less. In addition, it is necessary to choose different treatment methods according to different symptoms and signs, including nonsurgical treatment and surgical treatment. After strict conservative treatment, most patients can be relieved or cured, and only a small number of patients require further surgical treatment. After various experiments and clinical studies, the diagnosis and surgical methods of this disease are gradually improved, and there has been great development and innovation [4, 5].

The treatment of lumbar disc herniation can be divided into conservative treatment and surgical treatment. According to the natural course of lumbar disc herniation, conservative treatment is first required, unless there is serious nerve damage (such as decreased muscle strength and cauda equina syndrome).

In addition, surgical treatment can be divided into open surgery and minimal surgical intervention. Laparotomy usually involves removing the pulcossus core from the spinal disc by mediation, including normal laboratory nuclear and microscopic lumbar disc. This method is effective but causes great damage to the stability mechanism of the spine. For massive soft tissue injury and extensive bleeding, the nerve should be pulled during surgery, resulting in nerve injury and postoperative welding. For bleeding and rapid recovery, patients and doctors are taking it more and more. Below this, the spinal cord was removed in only one part of the area of the normal load, and there was no instability at the oval level of the spine.

Studies have shown that more than 90% of LDH patients have L3-S1 in the space between the lesions. Few (approximately 2%) of these patients require surgery due to poor conservative treatment effects. However, my country is a traditional agricultural country, and patients undergoing surgery for intervertebral disc herniation are still an important group. After decades of development, surgical treatment of lumbar intervertebral disc herniation can be divided into minimally invasive surgery and traditional open surgery. Traditional open surgery has a good surgical field of vision. Open surgery can make nerve decompression more thorough and have better and reliable surgical results [6, 7].

Among them, surgical treatment includes these categories. The first is anterior and posterior lumbar discectomy. The operation also requires the operator to have superb surgical skills, and the success rate of the operation can reach 90%. It has these advantages: it does not expose the spinal canal, does not touch the dura or nerve roots during the operation, and avoid harmful inflammation; it can also prevent scars, adhesions or bruises around the epidural and nerve roots. In addition, this method of operation will not be damaged. The structure behind the spine can prevent complications such as postoperative lumbar instability and spondylolisthesis, allowing patients to exercise their lower limbs and walk as soon as possible. Anterior direct vision lumbar discectomy also has many disadvantages, such as the inability to evaluate the herniated disc under direct vision, and the inability to remove the posterior disc, which can lead to nerve, peritoneal, and blood vessel damage. Posterior discectomy is currently the most common treatment in junior clinics.

The second type is percutaneous discectomy. This type of surgery has less trauma, quick recovery, does not affect the structure of the spinal canal, and does not affect the stability of the spine. According to foreign reports, the success rate is 85%. Because the operation is performed under online fluoroscopy, it has an additional injection effect on the operator, and the intervertebral disc cannot be completely removed or decompressed, causing spinal canal stenosis and accelerating spinal joint degeneration. It is limited to the clinical treatment of simple and acute disc herniation.

The third type is arthroscopic discectomy. It is a new surgical technique with minimal trauma, small surgical incision, less pain for the patient, high surgical tolerance, quick postoperative recovery, low psychological pressure on the patient, and does not affect the spinal canal structure, spinal stability, and does not affect the height of the intervertebral space. It has high precision and can effectively remove the nucleus pulposus, but the equipment required for this operation is expensive. Surgical intervention under endoscopy is technically very difficult, and surgeons must receive surgical training, that is, perform very strict and high-intensity exercises.

The fourth type is single-segment lumbar discectomy. The advantages of this kind of surgery are easy to use, safe, and less traumatic. Due to the short application time and the large amount of clinical operations, long-term follow-up is required to determine the curative effect and long-term complications, so a large amount of nucleus pulposus diseased tissue can be removed. The spinal cord changes before, during, and after lumbar discectomy are shown in Figure 1.

The fifth type is percutaneous endoscopic discectomy. This surgical method uses instruments and instruments to combine from the posterior surface to remove the protruding nucleus pulposus tissue through the “safety triangle” of the intervertebral foramen, thereby decompressing and loosening the nerve roots and spinal cord. This is a surgical method. For endoscopic or arthroscopic visualization surgery, Its advantages are as follows: it can completely remove the protruding lesions and nucleus pulposus directly, enter the intervertebral foramen to decompress, and completely loosen the compressed nerve roots and quickly and accurately give the operator the feeling of touching the nerve roots to prevent damage to the nerve roots [8, 9].

Among them, the key to improving surgical efficiency and long-term curative effect lies in the following: (1) a clear diagnosis and precise positioning, (2) understand the indications for surgery, (3) strictly follow the surgical procedures, and (4) pay attention to postoperative scientific rehabilitation training.

### 2.2. Lumbar Discectomy and Related Research

The most common cause of lumbar disc herniation is the disease of the nucleus pulposus tissue. Due to various reasons (physical damage, degeneration, etc.), the annulus fibrosus is damaged, the nucleus pulposus is prolapsed or detached, and the nerve roots around the prolapsed tissues have symptoms such as low back pain, numbness, and mechanical irritation. Chemical stimulation from the nucleus pulposus tissue can cause local inflammation, leading to radiculitis, cauda equina nerve damage, and other pathological changes.

The connective tissue of the nucleus pulposus of the lumbar intervertebral disc is composed of the neck, shoulder margin, and lumbar vertebral body. It is the main organ of the lumbar area. It not only plays an important role for the patient but also has a close influence on other parts. At present, a lot of research has been done on this aspect at home and abroad. Among them, high-incidence patients will use high-incidence lesions to relieve their pain when they have waist injuries and pain symptoms during application. At the same time, due to the existence of the lumbar intervertebral disc nucleus, the pelvis and neck dysfunction, joint deformities, and shoulder weakness occurred.

The main pharmacological effects of the lumbar intervertebral disc nucleus pulposus are to prevent osteoporosis, protect nerve tissue, promote blood circulation, and enhance the body's immunity. The protrusion of the nucleus pulposus of the lumbar intervertebral disc leads to poor stability and easy collapse, which affects the life of the patient. Therefore, in clinical treatment, research on preventive measures for lumbar disc herniation has become a current research hotspot.

The lumbar intervertebral disc nucleus pulposus is an important organ in the neck, shoulder, and lumbar muscles and has a great influence on its mechanical properties and functions. In the traditional research process, many scholars have conducted a large number of related experiments from different angles. For example, by observing the degree of flexion between the various parts of the patient's lumbar intervertebral disc and the change in the ratio of the internal cervical pressure to the outer diameter to determine whether there is injury, or determining the vertebral body pressure by measuring the thickness of the X-ray film, the distribution of stomata, and the size of the stomata, and use it as one of the basis for judging the location of the lesion and the nature of the lesion.

The main function of the lumbar intervertebral disc nucleus is to maintain the integrity of the vertebral body and pelvis, protect and repair the damaged surface, but because the patient's waist, back and other parts bear a large load, and long-term high-intensity exercise may easily lead to shoulder joint wear intensify.

Lumbar intervertebral disc nucleus extraction is mainly performed by effectively compacting, blessing, and wrapping the functional parts of the patient's waist and shoulders in the pelvis. The success of lumbar intervertebral disc nucleus extraction is closely related to the patient's bed rest and before and after the operation, and it is also a factor that affects the effect of rehabilitation treatment.

The trauma of traditional surgical treatment of patients with lumbar disc herniation is mainly reflected in the large surgical incision and the use of paraspinal muscles. Tools such as electrosurgery and bone removal performed more dissections. Articular process resection and blade resection have greater damage to the soft tissue and bone structure of the waist, and postoperative recovery is slower. Endoscopic nucleus pulposus ablation surgery helps to avoid soft tissue and bone damage, while exposing the surgical field of vision. Surgery is less traumatic and easier for patients to accept. The surgical procedure of lumbar discectomy is shown in Figure 2.

### 2.3. Study on the Stability of Lumbar Spine Segments

Related researchers believe that low back pain is mainly due to changes in mechanical factors during lumbar degeneration, that is, lumbar spine instability leads to low back pain symptoms and then put forward the concept of lumbar segmental stability.

There are still many controversies surrounding the definition and clinical diagnosis of segmental lumbar spine. The coexistence of several standards or evaluation theories may explain some instability, but there is a lack of consistent and comprehensive clinical diagnostic criteria to guide clinical work.

Some researchers believe that the two vertebral bodies and the adjacent intervertebral discs, facet joints and ligaments, back muscles and other structures maintain normal physiological activities and vertebral body stability. The stability of the spine reflects the relationship between the load and the displacement of the spine under its influence. Under the same load, the smaller the displacement of the moving parts, the greater the stability. Instead, the following applies: the greater the deviation, the worse the stability. It is also believed that the stability of the normal lumbar spine is maintained by intervertebral discs, facet joints, and ligaments and is affected by surrounding factors such as muscles, nerves, and abdominal pressure.

Under normal physiological pressure, the motion sequence and stability of the lumbar vertebrae are mainly achieved through the following aspects: the lumbar intervertebral disc maintains the range of motion between the vertebral bodies, and the small joints determine the direction of motion between the vertebral bodies. When the facet joint approaches the sagittal position, the vertebral body moves slightly forward; when the facet joint approaches the horizontal plane, the rotation range of dorsiflexion increases. The elasticity of the intervertebral discs, especially the annulus fibrosis, is an important factor in limiting the abnormal movement between the body's endplates. Ligaments help prevent excessive flexion, rotation, or displacement. When the ligamentum flavum is in the middle position, preloading the intervertebral disc helps to provide internal support for the spine. Facet joints play an important role in preventing extension, rotation, and forward movement. The lower back muscles also play an important role in the stability of the lumbar spine [10, 11].

Based on the mechanical relationship between stress and displacement, some researchers have proposed that lumbar instability refers to abnormal pressure, movement or pressure on the spine under normal pressure. This concept simply understands and defines the instability of the lumbar spine from mechanical factors, which ignores the complete factors such as spinal cord, nerves and blood vessels. Frymoyer proposed the definition of segmental instability of the lumbar spine: After a segment of the spine loses its rigidity, external force causes the segment to move more than the normal structure, which in turn leads to pain, pressure and potential nerve damage.

Under normal physiological pressure, any structure of the spine can maintain its normal positional relationship with the vertebral body without damaging or irritating the spinal cord or nerve roots of the spine. This is called clinical stability. Loss of this function is called clinically unstable. Mechanical instability refers to the stress exerted on the spine to study the relationship between the two, while clinical instability refers to the decrease in the stiffness of the active segment and the increase in the degree of mobility in biomechanics, compared with the normal structure of the spine. It is biomechanically unstable. There is a big change under the action. Clinically, excessive activity of the unstable spine can cause pain, and the underlying deformity of the spine can cause compression, irritation, or damage to the spinal cord or spinal cord nerve tissue. Therefore, the current clinical definition of lumbar spine instability is that the structure of the lumbar spine cannot maintain a normal positional relationship with the vertebral body under physiological pressure, resulting in loss or irritation of the spine.

After the sagittal plane of the lumbar spine loses its stability, under the action of physiological stress, the lumbar spine segment cannot maintain a normal positional relationship with the vertebral body, resulting in displacement, thereby increasing the neutral zone of lumbar spine mobility.  Table 1 shows the total NEMG value of each trunk muscle group clockwise.

The stability of the sagittal plane of the lumbar spine depends on the spine itself and the associated muscles. Lumbar instability due to system function or organ disease and injury, certain methods should be used to maintain stability. After the corresponding surgery, attention should be paid to the training of the muscles of the lower back to increase the strength of the spine, muscles, and ligaments of the lower back and enhance the stability of the sagittal plane of the lumbar spine [12–15].

## 3. Questionnaire and Research

### 3.1. Questionnaire Design Process

The subjects of the questionnaire survey were patients who had suffered from lumbar disc herniation and had undergone surgery. Through the distribution of online questionnaires or paper questionnaires, the collection and quantitative analysis of the information filled in by users are carried out to draw conclusions of the questionnaire.

1. In the preliminary preparation of the questionnaire, the number of questions should be as concise as possible to avoid fatigue of the interviewees
2. The questionnaire is released. The questionnaires were distributed through online questionnaires, on-site questionnaires, and inviting friends to help ask friends and students around them to fill in the questionnaires. A total of 170 questionnaires were distributed and 142 valid questionnaires were returned. The questionnaire recovery rate was 83.5%. The questionnaire distribution method and the results of the collection are shown in Table 2

(3) Questionnaire analysis. Organize the collected questionnaire information to get the required information data. The results of the questionnaire were analyzed. The results of the analysis included the degree of postoperative pain and the sagittal displacement of the lumbar spine of the postoperative patient. Some of the results obtained from the questionnaire are as follows

### 3.2. Questionnaire Survey Content

The first part is to select patients after lumbar intervertebral disc nucleus extraction, and investigate the postoperative pain degree of their waist and legs, walking, standing, and sleeping.

The second part compares the conditions of patients who have undergone single-segment lumbar disc nucleus extraction, conventional lumbar disc nucleus extraction, and cartilage plate curettage and analyzes the postoperative lumbar segmental sagittal displacement.

The third part is to sort out the information collected by the questionnaire to understand the degree of postoperative pain and the sagittal displacement of the lumbar spine of the postoperative patient. Part of the questionnaire survey results are as follows.

### 3.3. Analysis of the Reliability and Validity of the Questionnaire

Reliability and validity testing is a very important link in the process of empirical research, which is used to ensure the quality of the questionnaires used in survey research. Only when the measurement tool (i.e., questionnaire) meets the reliability and validity requirements, the research results can be convincing. Questionnaire reliability refers to the reliability of the survey, which reflects the stability and consistency of the results measured by measuring instruments or scales. The higher the reliability of the questionnaire, the lower the standard error of its measurement. Questionnaire validity is the basis to ensure that the research scale can truly reflect objective facts, is the basic condition of empirical research and has an important impact on the availability and accuracy of research results. The specific calculation method is shown in

(1) $$\begin{array}{c} \varpi_{a}=\frac{{\left(\sum \rho \right)}^{2}}{\left[{\left(\sum \rho \right)}^{2}+\sum \left(\phi \right)\right]}, \end{array}$$

(2) $$\begin{array}{c} \varpi_{b}=\frac{\left(\sum \rho^{2}\right)}{\left[\left(\sum \rho^{2}\right)+\sum \left(\phi \right)\right]}. \end{array}$$

Among them, *ϖ*_*a*_ is the combined reliability, *ϖ*_*b*_ is the average extraction variance, *ρ* is the standardized factor loading of the observed variable on the latent variable, and *ϕ* is the measurement error variance of the observed variable.

## 4. Analysis and Discussion

### 4.1. Analysis of Postoperative Pain Degree of Patients

In this questionnaire survey, patients who had undergone lumbar disc nucleus removal were selected to investigate their waist and leg conditions, walking, standing, and sleeping postoperative pain levels. The survey results are shown in Table 3.

It can be seen from Figure 3 that the proportion of respondents experiencing abnormal pain in different states after surgery was 0.05, 0.09, 0.03, and 0.01, respectively. It can be seen that most patients experience less abnormal pain after the operation, indicating that the operation has a certain effect on the treatment of the disease, and there are fewer abnormalities after the operation.

### 4.2. Analysis of the Postoperative Patients' Lumbar Segmental Sagittal Plane Displacement

By comparing the conditions of patients who had undergone single-segment lumbar disc nucleus extraction, conventional lumbar disc nucleus extraction, and cartilage plate curettage, the postoperative lumbar segment sagittal displacement was analyzed. The displacement situation is shown in Table 4.

It can be seen from Figure 4 that after a single-segment lumbar intervertebral disc nucleus extraction, the displacement values of the sagittal plane of the lumbar vertebrae segment were 0.05, 0.01, and 0.01, respectively, under the conditions of walking, sleeping, heavy physical work, and light physical work (0.2, 0.11 mm). It can be seen that, compared with other operations, single-segment lumbar discectomy is more stable in the sagittal plane of the lumbar spine within the physiological load range, and there is less displacement. The displacement may be caused or influenced by heavy load factors such as manual labor.

## 5. Conclusion

Lumbar disc herniation is a common disease, and many people are affected by it. It is a series of clinical manifestations caused by degeneration, rupture, and bulging of lumbar intervertebral discs caused by various factors, and compression of adjacent nerve roots or cauda equina. Among them, surgery is one of the methods to treat this disease, and lumbar discectomy is one of the typical representatives. However, there are still some patients whose body organs such as lumbar spine joints have also been badly affected after the operation. Therefore, this article carried out a basic study on the effect of single-segment lumbar disc nucleus extraction on the stability of the lumbar segmental sagittal plane. After a certain amount of experimental investigation and analysis, this article came to the conclusion that compared with other operations, after a single-segment lumbar disc nucleus extraction, the sagittal plane of the lumbar spine is relatively stable within the physiological load range, and the displacement occurs. In rare cases, the occurrence of displacement may be affected by heavy load factors such as physical labor. Moreover, most patients rarely experience abnormal pain after surgery, indicating that the surgery has a certain effect on the treatment of the disease, and there are fewer abnormalities after surgery.

## Figures and Tables

**Figure 1:** Spinal cord changes before, during and after lumbar discectomy.

**Figure 2:** Surgical procedure of lumbar discectomy.

**Figure 3:** Analysis of postoperative pain degree of patients.

**Figure 4:** Analysis of sagittal displacement of lumbar spine segments in postoperative patients.

**Table 1:** Clockwise total NEMG value of each trunk muscle group.

Trunk muscle groups	LSI	Non-LSI	Control
Total NEMG of left flexor	0.21 ± 0.019	0.26 ± 0.12	0.14 ± 0.072
Right flexor total NEMG	0.23 ± 0.034	0.19 ± 0.064	0.14 ± 0.062
Total NEMG of left extensor muscle	0.19 ± 0.064	0.22 ± 0.086	0.16 ± 0.059
Right extensor total NEMG	0.16 ± 0.081	0.13 ± 0.061	0.20 ± 0.089

**Table 2:** Questionnaire distribution method and collection results.

Questionnaire distribution method	Number of questionnaires issued	Number of questionnaires returned	Recovery rate (%)
Internet questionnaire	50	39	78
On-site questionnaire	80	72	90
Email	40	31	77.5

**Table 3:** Analysis of postoperative pain degree of patients.

Project	Normal	Slight pain	Moderate pain	Abnormal pain
Waist and leg condition	0.65	0.2	0.1	0.05
Walking condition	0.61	0.18	0.12	0.09
Standing condition	0.67	0.2	0.1	0.03
Sleeping condition	0.7	0.16	0.13	0.01

**Table 4:** Analysis of sagittal displacement of lumbar spine segments in postoperative patients.

Project	Walking condition	Sleeping condition	Heavy work	Light work
Single-segment lumbar discectomy	0.05	0.01	0.2	0.11
Routine lumbar discectomy	0.08	0.03	0.3	0.23
Cartilage scraping surgery	0.1	0.04	0.32	0.25

## Data Availability

The data underlying the results presented in the study are available within the manuscript.
